The article "Role of Activated Rac1/Cdc42 in Mediating Endothelial Cell Proliferation and Tumor Angiogenesis in Breast Cancer" was retracted in 2020. Reasons: duplicated images; original data or images not available; concerns about the data.

# Role of Activated Rac1/Cdc42 in Mediating Endothelial Cell Proliferation and Tumor Angiogenesis in Breast Cancer

**DOI:** 10.1371/journal.pone.0066275

**Published:** 2013-06-04

**Authors:** Ji Ma, Yan Xue, Wenchao Liu, Caixia Yue, Feng Bi, Junqing Xu, Jian Zhang, Yan Li, Cuiping Zhong, Yan Chen

**Affiliations:** 1 Department of Oncology, Xijing Hospital, The Fourth Military Medical University, Xi’an, Shannxi, China; 2 Department of Breast Surgery, Lanzhou General Hospital of People's Liberation Army, Lanzhou, Gansu, China; 3 Laboratory of Signal Transduction and Molecular Targeted Therapy, West China Hospital, Sichuan University, Chengdu, Sichuan, China; 4 Department of Radiology, Xijing Hospital, The Fourth Military Medical University, Xi’an, Shannxi, China; 5 Department of Biochemistry and Molecular Biology, Fourth Military Medical University, Xi’an, Shannxi, China; 6 Department of Ear Nose Throat Surgery, Lanzhou General Hospital of People's Liberation Army, Lanzhou, Gansu, China; University of Illinois at Chicago, United States of America

## Abstract

Angiogenesis is a well-established target in anti-cancer therapy. Although vascular endothelial growth factor (VEGF)-mediated angiogenesis apparently requires the Rho GTPases Rac1 and Cdc42, the relevant mechanisms are unclear. Here, we determined that activated Rac1/Cdc42 in MCF-7 breast cancer cells could decrease p53 protein levels and increase VEGF secretion to promote proliferation and tube formation of human umbilical vein endothelial cells (HUVECs). However, these effects are reversed after ubiquitin-proteasome breakage. In exploring potential mechanisms for this relationship, we confirmed that activated Rac1/Cdc42 could enhance p53 protein ubiquitination and weaken p53 protein stability to increase VEGF expression. Furthermore, in a xenograft model using nude mice that stably express active Rac1/Cdc42 protein, active Rac1/Cdc42 decreased p53 levels and increased VEGF expression. Additionally, tumor angiogenesis was inhibited, and p53 protein levels were augmented, by intratumoral injection of the ubiquitin-proteasome inhibitor MG132. Finally in 339 human breast cancer tissues, our analyses indicated that Rac1/Cdc42 expression was related to advanced TNM staging, high proliferation index, ER status, and positive invasive features. In particular, our data suggests that high Rac1/Cdc42 expression is correlated with low wt-p53 and high VEGF expression. We conclude that activated Rac1/Cdc42 is a vascular regulator of tumor angiogenesis and that it may reduce stability of the p53 protein to promote VEGF expression by enhancing p53 protein ubiquitin.

## Introduction

Tumor angiogenesis represents one of the most important pathological mechanisms in tumor growth, metastasis and recurrence [1], [2]. The treatment of tumor angiogenesis is impaired by its complicated and poorly understood pathogenesis. Until now, the main targeted inhibitor of tumor angiogenesis is bevacizumab, an inhibitor of vascular endothelial growth factor (VEGF). While the early success of anti-VEGF therapy in cancer patients is certainly encouraging, the effects of long-term VEGF inhibition will require close monitoring [3].

Tumor angiogenesis is initiated through the disruption of the balance of angiogenesis promoters and inhibitors [4]. As the most powerful angiogenesis promoter, VEGF plays a critical role in the development and maintenance of tumor vasculature and is regulated by classic signaling pathways, including the PI3K/AKT, Ras/MAPK and FAK/paxillin pathways [5], [6]. Moreover, accumulating evidence confirms that there are other key signaling molecules involved in tumor angiogenesis that regulate VEGF expression. A number of studies have indicated that some Rho guanosine triphosphatase (GTPase) family members are involved in tumor angiogenesis [7], [8]. Our previous findings demonstrated that in human breast cancer specimens, not only was high RhoA expression correlated with high VEGF expression, but RhoA can also increase VEGF expression to promote angiogenesis through an interaction with Murine Double Minute2 (MDM2) protein [9], [10]. In addition, other members of the Rho GTPase family Rac1 and Cdc42 also have significant effects on angiogenesis. Active Rac1 has been demonstrated to improve pathologic VEGF neovessel architecture and reduce vascular leak [11]. In addition, Rac1 signaling has been implicated in VEGF-mediated angiogenesis [12], [13]. Cdc42 reportedly participates in the processes of endothelial cell proliferation, migration and invasion [14], [15]. Although Rac1/Cdc42 signaling has been implicated in angiogenesis regulation, a comprehensive analysis of clinical data and the specific mechanisms by which Rac1/Cdc42 mediates VEGF-induced angiogenesis remain to be elucidated.

In our previous study, we observed that the disruption of Rac1 or Cdc42 expression results in up-regulation of p53 and down-regulation of VEGF [16]. In addition, p53 inhibited VEGF expression and thus affected angiogenesis development by regulating specificity protein-1(Sp1) and v-src sarcoma viral oncogene homolog (src) kinase activity [17]–[19]. Notably, some indications have emerged that activated Cdc42 can protect the epidermal growth factor receptor (EGFR) from ubiquitin degradation [20]. Furthermore, Rac1 regulated participation of the ubiquitin-ligase Skp2 in the cell proliferation process [21]. These findings suggest that activated Rac1/Cdc42 regulates some target molecules by affecting protein stability. Given this evidence, we hypothesized that activated Rac1/Cdc42 participates in VEGF-dependent tumor angiogenesis by increasing the degradation of angiogenesis inhibitors, including the p53 protein.

In the present study, we used MCF-7 human breast cancer cells, which express wild-type p53, a nude mouse model of breast cancer, and human breast cancer specimens to verify this hypothesis. We observed the effects of inhibiting the ubiquitin-proteasome pathway on HUVEC proliferation, tube formation, and the specific molecular mechanism induced by activated Rac1/Cdc42. Furthermore, in human tissue specimens, we analyzed the correlation of Rac1/Cdc42 with clinical features and angiogenesis factors. The results indicate that Rac1/Cdc42 is a vascular regulator involved in tumor angiogenesis, and that it may reduce the stability of p53 protein to increase VEGF levels by enhancing p53 protein ubiquitination. Our results indicate a novel molecular mechanism for tumor angiogenesis.

## Results

### Effect of MG132 on HUVEC proliferation and tube formation induced by activated Rac1/Cdc42

To observe whether Rac1/Cdc42 participates in tumor angiogenesis, the effects of activated Rac1/Cdc42 in MCF-7 cells on HUVEC proliferation and tube formation were examined. The constitutively activated Rac1 plasmid (V12Rac1) and Cdc42 plasmid (L61Cdc42) were used to produce activated Rac1 or Cdc42; pCEFL-GST served as the control plasmid. HUVECs were incubated with conditioned medium from MCF-7 cells stably transfected with one of these plasmids. After 24 h, the changes in HUVEC proliferation were not very obvious. However, after 48 h, the proliferation rates differed among the different groups. Compared to the control group, the medium derived from V12Rac1 or L61Cdc42–MCF-7 cells promoted HUVEC proliferation. Moreover, after treatment with the ubiquitin-proteasome inhibitor MG132, this increased effect was significantly inhibited (Fig. 1A). In the tube formation assay, HUVECs induced by V12Rac1– or L61Cdc42–MCF-7 cells associated with one another and formed more microtubes than did the control group. After MG132 treatment 48 h, however, the number of tubes formed by HUVECs induced by media from V12Rac1– or L61Cdc42–MCF-7 cells was reduced significantly (Fig. 1B and 1C). These results indicated that activated Rac1/Cdc42 in MCF-7 cells can accelerate HUVEC proliferation and tube formation to promote angiogenesis, and that these effects were partly inhibited by MG-132. However, the specific mechanism of angiogenesis induced by activated Rac1/Cdc42 needs to be further investigated.

**Figure 1:** Effect of MG132 on HUVEC proliferation and tube formation induced by active Rac1/Cdc42. The MTT and tube formation assays were performed as described in Material and Methods. (A) HUVECs were grown to confluence and were then cultured in preconditioned media (derived from GST–MCF-7, V12Rac1–MCF-7 and L61Cdc42–MCF-7 cells pretreated or not with MG132 for 12 h) for 24 h or 48 h; the GST–MCF-7 group was used as a control. (B) HUVECs were plated on Matrigel and incubated with the different preconditioned media for 6 h. Photographs were taken in five random power fields (200 ×). (C) Tube lengths were measured with Image-Pro Plus software. Histograms represent quantification of the HUVEC. The GST–MCF-7 group was used as a control. All data are expressed as mean ± standard deviation (SD) for three independent experiments. Statistical significance was assessed using one-way ANOVA and Student's *t*-test. *P<0.05, **P<0.01, for the GST–MCF-7 group vs the V12Rac1– or L61Cdc42– MCF-7 group. #*P*<0.05, ##*P*<0.01, for the MG132-added group vs the no-MG132 group.

### Activated Rac1/Cdc42 regulates p53 expression to affect VEGF expression in MCF-7 cells

To investigate whether p53 and VEGF are regulated by Rac1/Cdc42, the protein expressions of p53 and VEGF were measured in MCF-7 cells transfected with siRac1, V12Rac1, siCdc42 or L61Cdc42. Western blot results showed p53 expression to be increased in siRac1/Cdc42 groups, but decreased in V12Rac1/L61Cdc42 groups. At the same time, VEGF expression was reduced in the siRac1/Cdc42 groups, but augmented in the V12Rac1/L61Cdc42 groups (Fig. 2A–D). To further confirm whether p53 was regulated by Rac1/Cdc42 to affect VEGF expression, we used small interfering RNA of *Rac1/Cdc42* and *p53* (sip53) or *V12Rac1/L61Cdc42* and wild type *p53* (wt-p53) to transfect MCF-7 cells at the same time. Western blot results showed that although siRac1/Cdc42 could increase p53 and inhibit VEGF expression, reduced expression of VEGF caused by siRac1/Cdc42 disappeared after *p53* knockdown (Fig. 2E and 2G). Moreover, V12Rac1/L61Cdc42 could decrease p53 and augment VEGF expression, but up-regulated VEGF caused by V12Rac1/L61Cdc42 was attenuated after p53 over-expression (Fig. 2F, H). These assays indicate that the effect of Rac1/Cdc42 on VEGF was at least partly mediated by p53.

**Figure 2:** Rac1/Cdc42 regulates p53 expression to affect VEGF expression in MCF-7 cells. (A–D) MCF-7 cells were transfected with Rac1/Cdc42 small-interfering RNA (siRac1/Cdc42) or with negative control siRNA and with the plasmid pCEFL-GST-V12Rac1 (V12Rac1), pCEFL-GST-L61Cdc42 (L61Cdc42) or pCEFL-GST-neo using lipofectamine 2000 for 48 h. Protein and RNA were then extracted and subjected to western blot analyses. Total protein was subjected to 15% SDS-PAGE; membranes were incubated with anti-Rac1, anti-Cdc42, anti-p53, anti-VEGF, or anti-β-actin antibody. (E–H) MCF-7 cells were transfected with siRac1/Cdc42 or with p53 siRNA (sip53) and either activated Rac1/Cdc42 plasmid (V12Rac1/L61Cdc42) or wild-type p53 expression plasmid (wt-p53) with lipofectamine 2000 for 48 h. Protein was then extracted and subjected to 15% SDS-PAGE; membranes were incubated with anti-p53, anti-VEGF, or anti-β-actin antibody. The data represent three independent experiments.

### Activated Rac1/Cdc42 promotes ubiquitin-mediated degradation of p53 to increase VEGF production in MCF-7 cells

Given that the amount of p53 protein could be modified by changes in the rate of synthesis or degradation [22], we hypothesized that Rac1/Cdc42 affected degradation of p53. To test this hypothesis, the ubiquitin-proteasome inhibitor MG-132 was utilized to analyze p53 protein levels. Western blot results revealed that p53 protein was inhibited by V12Rac1/Cdc42, but a large accumulation of p53 protein was observed in the presence of V12Rac1/Cdc42, together with MG-132 (Fig. 3A). Additionally, immunoprecipitation data showed that V12Rac1/Cdc42 could reduce p53 protein levels and increase the amount of ubiquitinated p53 (Fig. 3B). The VEGF ELISA assay also showed that in MCF-7 cells, V12Rac1/LCdc42 increased VEGF secretion after 24 h and 48 h, compared to the control group. However, VEGF expression induced by V12Rac1 or L61Cdc42 decreased after treatment with MG132 (Fig. 3C). These results confirmed that active Rac1/Cdc42 affected and promoted ubiquitin-mediated degradation of p53 to increase VEGF production.

**Figure 3:** Effect of MG132 on VEGF and p53 expression induced by active Rac1/Cdc42. (A) GST–MCF-7, V12Rac1–MCF-7, and L61Cdc42–MCF-7 cells were incubated, and MG132 was added to select samples for 12 and 24 h, respectively. After incubation, the media were analyzed for VEGF levels using ELISA assay; cell numbers were counted. Data are expressed as the mean ± standard deviation (SD) for three independent experiments. Statistical significance was assessed with one-way ANOVA and Student's t-test. *P<0.05, **P<0.01, for the GST–MCF-7 group vs V12Rac1– or L61Cdc42–MCF-7 group. #*P*<0.05, ##*P*<0.01, for the MG132-added group vs the no-MG132-added group. (B, C) MCF-7, GST–MCF-7, V12Rac1–MCF-7 and L61Cdc42–MCF-7 cells were incubated, and MG132 was added to select samples for 24 h. After incubation, the cells were analyzed by western blot assay. p53, p21 and β-actin expression was examined. β-actin protein levels were used as a loading control. (D) The immunoprecipitation assay was performed as described in Material and Methods. Total protein was extracted from MCF-7, GST–MCF-7, V12Rac1–MCF-7 and L61Cdc42–MCF-7 cells and subjected to an immunoprecipitation assay. p53 protein expression was examined. β-actin protein levels were used as a loading control.

### Effect of intratumoral injections of MG132 on vascularization induced by activated Rac1/Cdc42 in MCF-7 cell xenografts

To further evaluate the effects of MG132 on tumor angiogenesis induced by V12Rac1/LCdc42, we injected 10 mg/kg MG132 or PBS every 2 days into pre-established, MCF-7 breast tumors (approximately 200 mm^3^) grown in nude mice. Immunolabeling for VEGF was much higher in tumors excised from mice in the V12Rac1 and L61Cdc42 groups than in those from the control group (Fig. 4). Moreover, p53 expression was lower in the V12Rac1 and L61Cdc42 groups than in the blank or control groups. However, MG312 injections dramatically inhibited the increase in VEGF expression and enhanced the decrease in p53 expression in the V12Rac1 and L61Cdc42 groups compared with the control group. There was no significant difference between the blank and control groups. These data revealed that *in vivo*, MG132 could reverse the effects of activated Rac1/Cdc42 on p53 and VEGF expression to suppress tumor angiogenesis.

**Figure 4:** Effect of intratumoral injections of MG132 on vascularization induced by active Rac1/Cdc42 in MCF-7 cell xenografts. These experiments were described in the Materials and Methods section. Stably transfected cells (MCF-7, GST–MCF-7, V12Rac1–MCF-7, L61Cdc42–MCF-7) were used for xenografts in nude mice. When the tumors reached a volume of 200 mm3, the mice were treated with intratumoral injections of a specific dose of MG132 (10 mg/kg) or PBS. (A, B) Intratumoral vascularization was assessed by VEGF and p53 immunolabeling (400 × power) on paraffin-embedded MCF-7 cell tumor sections. Representative images are shown. Integrated optical density (IOD) values of VEGF and p53 protein expression were evaluated. ImagePro Plus software was used to analyze the IOD values of the positive areas of immunohistochemical staining. The resulting histograms are presented here. A statistical analysis was performed using a one-way ANOVA. The results are presented as mean ± SD for six mice. *P<0.05; **P<0.01.

### Relationship between Rac1/Cdc42 expression and clinical histopathologic characteristics in breast cancer specimens

To assess the significance of Rac1/Cdc42 protein expression in the development and progression of breast cancer, we compared histopathologic characteristics of tumors from 339 patients with available Rac1/Cdc42 protein status in breast cancer samples. The correlation of Rac1/Cdc42 protein expression with different clinical histopathologic factors is presented in Table 1. Statistically significant correlations were found between high Rac1/Cdc42 expression and advanced TNM staging (*P*<.001), proliferation index (Ki67 status; *P*<.001), ER status (*P*<.001), and positive invasive features, including lymph node metastasis (*P*<.001) and tumor invasion (*P*<.001) (Table 1). Correlation coefficients are presented in Table 2. However, Rac1/Cdc42 expression did not correlate with patient age, tumor size, histology differentiation or Her-2 status.

**Table 1:** Statistical results of Rac1/Cdc42 expression in 339 breast cancer specimens.

Variable		No.	Rac1 expression		*p*	Cdc42 expression		*p*
			Positive (%) Negative (%)			Positive (%) Negative (%)		
Age(years)					185^a^			.989^a^
≤ 50		141	105 (74.5)	36		87 (61.7)	54	
>50		198	(25.5)	65		(38.3)	76	
			133 (67.2)			122 (61.6)		
			(32.8)			(38.4)		
Tumor size					.280^a^			.311^a^
≤ 2 cm		142	95 (66.9)	47		83 (58.5)	59	
>2 cm		197	(33.1)			(41.5)		
			143 (72.6)	54		126 (64.0)	71	
			(27.4)			(36.0)		
TNM stage					<.0001^a^			<.0001^a^
I∼II		116	22 (19.0)	94		35 (30.2)	81	
III∼IV		223	(81.0)	79		(69.8)		
			144 (64.6)			128 (57.4)	95	
			(35.4)			(42.6)		
Lymph	node				<.0001^a^			<.0001^a^
Metastasis		228	195 (85.5)	33		184 (80.7)	44	
Positive		111	(14.5)			(19.3)	86	
Negative			43 (38.7)	68		25 (22.5)		
			(61.3)			(77.5)		
Histology					.464^b^			.621^b^
Poorly		105	75 (71.4)	30		68 (64.8)	37	
differentiated			(28.6)			(35.2)		
Moderately		106						
differentiated			78 (73.6)	28		66 (62.3)	40	
								
Well		128	(26.4)			(37.7)		
differentiated								
			85 (66.4)	43		75 (58.6)	53	
			(33.6)			(41.4)		
Tumor invasion					<.0001^a^			<.0001^a^
Yes		254	206 (81.1)	488		188 (74.0)	66	
No		85	(18.9)					
ER status			32(37.6)	53	<.0001^a^	21 (24.7)	64	
Positive		185	(62.4)			75.3		
Negative		154						
Her-2 status			90(48.6)		.237^a^	86(46.5)		.268^a^
Positive		68	95(51.4)			99(53.5)		
Negative		271	148(96.1)	6(3.9)		123(79.9)		
Ki67 status					<.0001^a^	31(20.1)		<.0001^a^
Positive		227	52(76.5)					
Negative		112	16(23.5)			46(67.6)		
			186(68.6)			22(32.4)		
			85(31.4)			163(60.1)		
						108(39.9)		
			184(81.1)					
			43(18.9)			169(74.4)		
			54(48.2)			58(25.6)		
			58(51.8)			40(35.7)		
						72(64.3)		

a The Fisher's exact test was used for statistical analyses. *P* values <0.05 were considered statistically significant.

b The Pearson's chi square test was used for statistical analyses.

**Table 2:** Correlation of Rac1/Cdc42 expression with clinical histopathologic characteristics in 339 breast cancer specimens.

Variable	Rac1 expression	*p* a	Cdc42 expression	*p* a
	Correlation coefficient (*r_s_*)		Correlation coefficient (*r_s_*)	
Age(years)	.079	.149	.001	.987
Tumor size	−.061	.260	−.056	.305
TNM stage	−.433	.0001	−.295	.0001
Lymph node metastasis	.480	.0001	0.562	.0001
Differentiated status	.049	.365	.053	.332
Tumor invasion	.412	.0001	.440	.0001
ER status	−.517	.0001	−.342	.0001
Her-2 status	.069	.208	.062	.257
Ki67 status	.338	.0001	.375	.0001

a The Spearman correlation test was used for statistical analyses. *P* values <0.05 were considered statistically significant.

### Correlation of Rac1/Cdc42 expression with wild-type p53 and VEGF expression in breast cancer specimens

Because the wild-type p53 is the functional form of the p53 protein, examining the level of this form is critical. To estimate the degree of correlation between Rac1/Cdc42 expression and wt-p53 and VEGF in the tumor specimens, we identified 145 specimens that expressed wt-p53 protein among the 339 breast cancer specimens by *p53* gene mutation analysis. The statistical analysis indicated that both Rac1 and Cdc42 protein expression were inversely correlated with wt-p53 expression (correlation coefficient [*r_s_*] = –.406, *P*<.0001; and *r_s_* = –.263, *P* = .001; respectively). In contrast, statistically significant positive correlations were observed between expressions of Rac1 and VEGF (*r_s_* = .268; *P* = .001) and between Cdc42 and VEGF (*r_s_* = .224; *P* = .007) (Table 3). These data indicate that high Rac1/Cdc42 expression is correlated with low wt-p53 expression and high VEGF expression.

**Table 3:** Correlation of Rac1/Cdc42 expression with wild-type p53 and VEGF protein in 145 breast cancer specimens containing the wild-type p53 protein.

Variable	No.	Rac1 Expression	*p* a		Cdc42 Expression		*p* a
		Positive (%) Negative (%)			Positive (%) Negative (%)		
wt-p53				<.0001^b^	30 (44.1)	38	.001^d^
Positive	68	29 (42.6)	39		(55.9)		
Negative	77	(57.4)			54 (70.1)	23	
					(29.9)		
		63 (81.8)	14				.007^e^
		(18.2)					
VEGF				.001^c^			
Positive	105	75 (71.4)	30		68 (64.8)	37	
Negative	40	(28.6)			(35.2)		
		17 (42.5)	23		16 (40.0)	24	
		(57.5)			(60.0)		

a The Spearman correlation test was used for statistical analyses. *P* values <0.05 were considered statistically significant.

b Correlation coefficient (*r_s_*) = −.406.

c *r_s_*  = .268.

d *r_s_*  = −.263.

e *r_s_*  = .224.

## Discussion

Although the *Rac1* and *Cdc42* oncogenes have been showed to promote carcinogenesis progression and angiogenesis, and to play critical roles in VEGF-dependent tumor angiogenesis [11]–[15], comprehensive clinical data and the specific mechanisms of Rac1/Cdc42-mediated tumor angiogenesis require further investigation. In the present study, we investigated the regulatory role of active Rac1/Cdc42 on p53 and VEGF *in vitro* and *in viv*o and investigated the correlation of Rac1/Cdc42 expression with tumor angiogenesis in breast cancer specimens. Our data indicate that Rac1/Cdc42 is the vascular regulator involved in tumor angiogenesis and that it may reduce the stability of p53 protein to promote VEGF expression by enhancing p53 protein ubiquitin.

Rac1/Cdc42 plays a key role in HUVEC proliferation and tube formation. Some studies indicate that silencing *Rac1/Cdc42* in HUVECs inhibits VEGF-mediated tube formation, cell migration, invasion and proliferation [28], [29]. Furthermore, endothelial-specific excision of Rac1/Cdc42 leads to defective development of vessels and embryonic lethality, supporting an essential role for Eac1/Cdc42 in vascular development [13], [30]. Coincident with these findings, our data demonstrate that activated Rac1/Cdc42 increased HUVEC proliferation and tube formation. In present study of angiogenesis, we focused on the effects of activated Rac1/Cdc42 in MCF-7 cells on HUVECs. Whatever the context of the study, VEGF remains the important factor affecting vascular endothelial cells. We believe that activating of Rac1/Cdc42 in cancer cells is a critical step in tumor angiogenesis to increase VEGF secretion and promote formation of primary vessels from vascular endothelial cells.

Recent studies suggest that Rac1/Cdc42 regulates its target molecule to participate in tumorigenesis through both gene transcription regulation and post-translational modification. Activated Cdc42 influences the interactions of the ubiquitin- ligase c-Cbl with the EGFR to protect the EGFR from ubiquitin degradation [20]. Furthermore, activated Rac1 increases the activity of the ubiquitin- ligase Skp2 protein by down-regulating p27 to promote cell proliferation [21]. In our previous study, we observed that disruption of Rac1 or Cdc42 expression results in up-regulation of p53 and down-regulation of VEGF [16], [31]. However, whether Rac1/Cdc42 affects p53 expression by ubiquitination remains unclear. In this study, activated Rac1/Cdc42 inhibited p53 and increased VEGF expression. Importantly, the inhibitory effects of activated Rac1/Cdc42 on p53 expression were reversed after MG132 treatment. Moreover, activated Rac1/Cdc42 was able to reduce p53 protein levels and increase the amount of ubiquitinated p53. These results suggest that Rac1/Cdc42 can regulate p53 protein by enhancing its degradation, thereby promoting VEGF expression. This finding represents a new insight into the mechanism of Rac1/Cdc42-mediated tumor angiogenesis; and suggests a novel strategy for tumor angiogenesis treatment. However, ubiquitin-proteasome inhibitor MG132 which is a kind of unspecific inhibitor could reverse some tumor suppressor protein levels in cancer cells to play the anticancer effects. In this study, using MG132 just indicated that active Rac1/Cdc42 in cancer cells may promote the degradation of antiangiogenesis factors through ubiquitin-proteasome pathway. Therefore, the specific ubiquitin molecule mediates this ubiquitination progression remains unclear and requires further investigation.

To date, studies examining the association of Rac1/Cdc42 and the clinical histopathologic characteristics of human breast cancer tissues are rare. Fritz *et al*. reported that in 50 breast cancer specimens, high Rac1 expression was significantly related to tumor histological grade and proliferation index, but not to Her-2 status [32]. Coincident with these findings, we examined Rac1/Cdc42 expression in 339 human breast cancer specimens and determined that high levels of Rac1/Cdc42 expression were correlated with advanced TNM staging and proliferation index (Ki-67 status) but not with Her2 status. However, the Fritz study did not indicate the relationship between Rac1/Cdc42 expression and other hormone status, or invasiveness. In our study, we found that high Rac1/Cdc42 expression was significantly correlated with lymph node metastasis, tumor invasion and low ER expression. Su *et al*. determined that as a modulator, active Rac1/Cdc42 decreased *ER* transcription, and that inhibition of Rac1/Cdc42 enhanced *ER* transcriptional activity in MCF-7 cells [33]. These findings are consistent with our data in human breast cancer specimens. Importantly, we observed that high Rac1/Cdc42 expression was correlated with low *wt-p53* expression and high *VEGF* expression in 145 specimens that expressed wt-p53. Although expression of Rac1/Cdc42 in breast cancer specimens has been investigated previously, to the best of our knowledge, the current report is the first comprehensive analysis of the regulatory relationship between these angiogenesis molecules in breast cancer tissues. The results of this study fully support our previous data collected *in vitro*.

Taken together, our data demonstrate that Rac1/Cdc42 signaling is critical in tumor angiogenesis; activated Rac1/Cdc42 reduces the stability of p53 protein to promote VEGF expression by enhancing p53 protein ubiquitin. Moreover, Rac1/Cdc42 is significantly correlated with metastasis, invasion and tumor angiogenesis in breast cancer and is a potential prognosis marker in breast cancer. Although the contribution of Rac1/Cdc42 to tumor angiogenesis is complicated and not yet fully understood, our findings provide further understanding and imply a novel target for tumor angiogenesis treatment.

## Materials and Methods

### Cell lines and reagents

The breast cancer cell line MCF-7 was obtained from the American Type Culture Collection (Rockville, Md) and was cultured according to the supplier's directions and guidelines. HUVECs were isolated, cultured, and characterized as previously described [22]. Cells were maintained at 37°C in a humidified incubator with 5% CO_2_. Mouse monoclonal anti-Rac1 (1∶1000 dilution; Abcam, Hong Kong, China), mouse monoclonal anti-Cdc42 (1∶1000 dilution; Abcam), mouse monoclonal anti-p53 (1∶500 dilution; Santa Cruz Biotechnology, Inc., Santa Cruz, California), rabbit monoclonal anti-p21 (1∶300 dilution; Santa Cruz Biotechnology), mouse monoclonal anti-ubiquitin (1∶300, Santa Cruz Biotech), rabbit polyclonal anti-VEGF (1∶1000 dilution; Cell Signaling, Danvers, Mass), rabbit polyclonal anti-β-actin (1∶3000 dilution; BIOS Biotechnology, Beijing, China), VEGF ELISA assay kit (R&D Corporation), Geneticin (G418, Invitrogen), protein G-sepharose (Sigma-Aldrich, St. Louis, Mo), and MG132 (Sigma-Aldrich, St. Louis, Mo) were used according to the manufactures' instructions.

### Gene transfection and stable transfected cells

The eukaryotic expression plasmids pCEFL-GST-neo control, pCEFL-GST-V12Rac1 and pCEFL-GST-L61Cdc42 (constitutively activated Rac1 and Cdc42) were generously provided by Professor Zheng Yi (University of Cincinnati, Cincinnati, USA). According to the manufacturer's instructions, MCF-7 cells were plated in a 6-well plate and grown overnight to 70–80% confluence without antibiotics. Cells were then transfected with Lipofectamine 2000 (Invitrogen, Carlsbad, California) and different plasmids. Five hours later, the transfection medium was replaced with DMEM supplemented with serum. The transfected cells were selected with 450 µg/ml G418 2 days after transfection. After 2 weeks, G418 was reduced to the maintenance dose of 300 µg/ml. After 4 weeks, these polyclonal, stable transfected cells were trypsinized and transferred to 10 cm tissue culture dishes. Monoclones were picked in a 6-well plate and expanded for an additional 2 months.

### MTT assay

HUVECs were plated at a density of 4 × 10^4^ cells/cm^2^ in 24-well plates in complete medium and allowed to adhere overnight. Stably transfected MCF-7 cells were cultured, and MG132 was added at a concentration of 2.5 µmol/L for 12 h. Conditioned culture medium from the stably transfected MCF-7 cells was subsequently placed in the HUVEC-containing wells; the whole plate was incubated in a culture chamber for 24 h or 48 h. HUVECs were then incubated for 4 h with MTT (3-(4,5-dimethylthiazol-2-yl)-2,5-diphenyl tetrazolium bromide). Formazan crystals thus formed were dissolved in 750 µl of dimethyl sulfoxide after the medium was aspirated. The solution was transferred to a 96-well plate, and optical density value was recorded at 570 nm on a microplate reader (Model 680, Bio-Rad, USA). The results are expressed relative to the OD value of HUVEC monocultures on day 1 of the assay.

### Tube formation assay

Sterile 24-well plates were coated with 200 µl Matrigel and incubated at 37°C for 1 h to form gels. After polymerization of the gels, 1.0 × 10^5^ HUVECs were seeded into each well and incubated with 1.0 ml DMEM containing 1% FBS. Stably transfected MCF-7 cells were then cultured, and MG132 was added at a concentration of 2.5 µmol/L for 48 h. Conditioned culture medium from the stably transfected MCF-7 cells was placed in the HUVEC-containing wells for 6 h in a culture chamber. Five different fields were chosen randomly in each well, and photographed. Lengths of the tubes were measured using Image-Pro Plus software (Media Cybernetics, L.P., Silver Spring, MD, USA) and were each expressed as total length (mm) per microscopic field for each well.

### ELISA assay

To assess VEGF secretion in the supernatants of the stably transfected cells, the cells were incubated in serum-free medium with 2.5 µmol/L MG132. After 24 or 48 h, the media were collected, centrifuged to remove cellular debris, and stored at −70°C until being assayed for VEGF. VEGF secreted in the culture medium was measured by ELISA according to the manufacturer's instructions. The data are expressed in pg of VEGF/10^5^ cells/ml.

### Western blot

MCF-7 cells were homogenized in RIPA lysis buffer, and insoluble material was removed by centrifugation at 4°C. From each sample, 80–100 µg of total protein extract was resolved by 12% SDS-PAGE and transferred to nitrocellulose membranes (Amersham Biosciences, Piscataway, NJ). The membranes were blocked in 5% milk and probed with the antibodies overnight at 4°C. The membranes were washed and incubated with a horseradish peroxidase (HRP)-conjugated secondary antibody (Santa Cruz Biotech) for 1 h at 37°C. Chemiluminescent HRP substrate solution (Millipore, USA) was used to develop the images.

### Immunoprecipitation assay

The immunoprecipitation assay was performed as described previously [23]. Cell lysates were incubated with an anti-p53 antibody. The immune- complexes were precipitated with protein A- or protein G-Sepharose 4B (Amersham Biosciences). After washing with lysis buffer, the precipitated proteins were separated by SDS-PAGE and transferred to nitrocellulose membranes (Amersham Biosciences). The blots were probed with anti-ubiquitin overnight at 4°C. A western blot analysis was then performed.

### Xenograft study in nude mice

For inoculation into nude mice, the stably transfected MCF-7 cells were washed with PBS, digested with trypsin, and resuspended in serum-free DMEM medium. After centrifugation (800 rpm), the cell pellets were resuspended in DMEM. The cell suspension (5 × 10^6^ cells in 100 µl of PBS) was injected subcutaneously into the hind legs of 4-week-old female BALB/C athymic (nu/nu) mice (SLAC Laboratory Animal Company, Shanghai, China)[10]. When tumors reached volumes of 200 mm^3^, the mice were arbitrarily assigned to different groups ((n = 6 each) to receive intratumoral injections of a specific dose of MG132 (10 mg/kg) or PBS. Intratumoral injections were repeated every 3 days for a total of 20 days. On day 20, the mice were sacrificed and their tumors were removed for analysis.

All of the experimental procedures were conducted in accordance with the Detailed Rules for the Administration of Animal Experiments for Medical Research Purposes issued by the Ministry of Health of China and received ethical approval by the Animal Experiment Administration Committee of the Fourth Military Medical University (Xi'an, P. R. China). All efforts were made to minimize the animals' suffering and to reduce the number of animals used.

### Immunohistochemistry

Immunohistochemical staining was performed to assess expression of VEGF and p53 proteins, as described previously [9]. For immunohistochemistry, formalin-fixed tumor tissues were embedded in paraffin, and serial 4- µm sections were obtained using a Leica microtome. For staining, tumor sections were dewaxed in toluene, rehydrated in an alcohol gradient, and permeabilized in citrate buffer (pH 6.0). To eliminate endogenous peroxidase activity, the tumor sections were incubated with 3% H_2_O_2_ for 5 min, washed in PBS, incubated overnight with different antibodies, and subsequently incubated with biotinylated goat anti-rat or anti-rabbit IgG antibody for 15 min. After washing, the sections were incubated with streptavidin-peroxidase, lightly counterstained with hematoxylin, and observed under a photomicroscope.

### Staining evaluation

This study was approved by the Clinical Trials Administration Committee and the Ethics Committee of the Fourth Military Medical University (Xi'an, P. R. China). All samples were obtained from the Tissue Bank of the Fourth Military Medical University Cancer Center and coded anonymously in accordance with local ethical guidelines. All patients agreed to participate in this study. Written informed consent was obtained from patients, and protocol was approved by the Review Board of Fourth Military Medical University Cancer Center. Fresh breast carcinoma specimens were collected from 339 female patients at the Xijing Hospital of the Fourth Military Medical University (Xi’an, China) and Lanzhou General Hospital of CPLA (Lanzhou, China) from 2006 to 2011. Genomic DNA from 339 tissue specimens was extracted for *p53* gene mutation analysis [24]. Rac1/Cdc42 expression was detected in all of the specimens, and *wt-p53* and *VEGF* expression was detected in 145 specimens containing wt-p53 protein. Tissue specimens were examined separately by two pathologists under double-blinded conditions without prior knowledge of the clinical status of the specimens. Molecule expression was scored as positive if >10% of the cells exhibited moderate to strong staining. Expression was scored as negative if either cytoplasmic or membranous staining was noted in <10% of the cells or if neither cytoplasmic nor membranous staining was observed [25]. The Ki67 immunohistochemistry results were reported as the percent positivity of neoplastic cells. For this analysis, we classified the Ki67 levels as negative if <16% or positive if ≥16% [26]. HER2 positivity was defined as 3+ staining on immunohistochemistry or an amplification ratio for fluorescent *in situ* hybridization if >2.2 [27].

### Statistical analysis

Experiments *in vitro* were performed in triplicate. Data from all quantitative assays are expressed as mean ± standard error and were analyzed statistically using a one-way ANOVA followed by Student's *t*-test. *P*<0.05 was considered statistically significant. In the *in vivo* study, associations between Rac1/Cdc42 expression and categorical variables were analyzed by the χ^2^ test or Fisher's exact test, as appropriate. Correlations between Rac1/Cdc42 expression and categorical variables were analyzed by the Spearman correlation test.
